RETRACTED

# FOXM1 modulates 5-fluorouracil sensitivity in cholangiocarcinoma through thymidylate synthase (TYMS): implications of FOXM1–TYMS axis uncoupling in 5-FU resistance

**DOI:** 10.1038/s41419-018-1235-0

**Published:** 2018-12-11

**Authors:** Kitti Intuyod, Paula Saavedra-García, Stefania Zona, Chun-Fui Lai, Yannasittha Jiramongkol, Kulthida Vaeteewoottacharn, Chawalit Pairojkul, Shang Yao, Jay-Sze Yong, Sasanan Trakansuebkul, Sakda Waraasawapati, Vor Luvira, Sopit Wongkham, Somchai Pinlaor, Eric W.-F. Lam

**Affiliations:** 1 Department of Surgery and Cancer, Imperial College London, Imperial College London, Hammersmith Hospital Campus, London, W12 0NN UK; 2 Biomedical Science Program, Graduate School, Khon Kaen University, Khon Kaen, 40002 Thailand; 3 Cholangiocarcinoma Research Institute, Khon Kaen University, Khon Kaen, 40002 Thailand; 4 Department of Biochemistry, Faculty of Medicine, Khon Kaen University, Khon Kaen, 40002 Thailand; 5 Department of Pathology, Faculty of Medicine, Khon Kaen University, Khon Kaen, 40002 Thailand; 6 Department of Surgery, Faculty of Medicine, Khon Kaen University, Khon Kaen, Thailand; 7 Department of Parasitology, Faculty of Medicine, Khon Kaen University, Khon Kaen, Thailand

## Abstract

Fluorouracil (5-FU) is the first-line chemotherapeutic drug for cholangiocarcinoma (CCA), but its efficacy has been compromised by the development of resistance. Development of 5-FU resistance is associated with elevated expression of its cellular target, thymidylate synthase (TYMS). E2F1 transcription factor has previously been shown to modulate the expression of FOXM1 and TYMS. Immunohistochemical (IHC) analysis revealed a strong correlated upregulation of FOXM1 (78%) and TYMS (48%) expression at the protein levels in CCA tissues. In agreement, RT-qPCR and western blot analyses of four human CCA cell lines at the baseline level and in response to high doses of 5-FU revealed good correlations between FOXM1 and TYMS expression in the CCA cell lines tested, except for the highly 5-FU-resistant HuCCA cells. Consistently, siRNA-mediated knockdown of FOXM1 reduced the clonogenicity and TYMS expression in the relatively sensitive KKU-D131 but not in the highly resistant HuCCA cells. Interestingly, silencing of TYMS sensitized both KKU-D131 and HuCCA to 5-FU treatment, suggesting that resistance to very high levels of 5-FU is due to the inability of the genotoxic sensor FOXM1 to modulate TYMS expression. Consistently, ChIP analysis revealed that FOXM1 binds efficiently to the TYMS promoter and modulates TYMS expression at the promoter level upon 5-FU treatment in KKU-D131 but not in HuCCA cells. In addition, E2F1 expression did not correlate with either FOXM1 or TYMS expression and E2F1 depletion has no effects on the clonogenicity and TYMS expression in the CCA cells. In conclusion, our data show that FOXM1 regulates TYMS expression to modulate 5-FU resistance in CCA and that severe 5-FU resistance can be caused by the uncoupling of the regulation of TYMS by FOXM1. Our findings suggest that the FOXM1–TYMS axis can be a novel diagnostic, predictive and prognostic marker as well as a therapeutic target for CCA.

RETRACTED

## Introduction

Opisthorchiasis, a hepatobiliary disease caused by infection with a small human liver fluke *Opisthorchis viverrini*, is a major health problem in Southeast Asia, predominantly in Thailand, Lao PDR, South Vietnam and Cambodia. *O. viverrini* infection has been proven to be associated with cholangiocarcinoma (CCA) development^1^. At least 6 million people are currently infected with *O. viverrini* and thus at risk for CCA^2^. Extensive research has revealed that *O. viverrini* infection induces inflammation, leading to periductal fibrosis and ultimately cholangiocarcinogenesis in patients^2–5^. Currently, surgical resection is the most effective treatment for operable cases but most CCA patients are inoperable^6,7^, resulting in poor prognosis. Despite chemotherapy, particularly with the first-line drug 5-fluorouracil (5-FU), resistance eventually develops over time^8–10^. Therefore, an understanding of the mechanism involved in the development of 5-FU resistance is urgently needed for predicting and for improving treatment efficacy.

Previous cDNA microarray studies have revealed the upregulation of Forkhead box M1 (FOXM1) mRNA levels in tumour specimens derived from *O. viverrini*-associated CCA patients^11^. FOXM1 is a potent oncogenic transcription factor involved in normal development and also progression of numerous cancer types^12^. Furthermore, FOXM1 is crucial for chemotherapeutic drug response and resistance in many cancers^13–15^ and is therefore an attractive target for therapeutic intervention^15^. Thymidylate synthase (TYMS) is an enzyme involved in DNA synthesis process. It catalyses the conversion of deoxyuridine monophosphate (dUMP) to deoxythymidine monophosphate (dTMP) and a target of 5-FU chemotherapy. Specifically, the active metabolite of 5-FU, fluorodeoxyuridine monophosphate (FdUMP) binds to the active site of for dUMP on TYMS, leading to the formation of an inactive FdUMP–TYMS complex and inhibition of the conversion of dUMP to dTMP. This causes deoxynucleotide (dNTP) pool imbalance and, ultimately, DNA damage and cell death^16^. Upregulation of *TYMS* gene has been reported following 5-FU treatment in human CCA cell lines^17^; however, its steady-state mRNA levels in human CCA tissues are not significantly correlated with the response to 5-FU^18^. Like FOXM1, the transcription factor E2F1 is a potent oncogene involved in cell cycle progression, DNA-damage response, drug resistance and apoptosis^19–21^. Both FOXM1 and TYMS have been reported to be the target genes of the E2F1 transcription factor^20,22–24^. Based on these previous findings, we therefore hypothesized that FOXM1 and E2F1 may coordinately modulate 5-FU sensitivity by targeting TYMS in CCA. Hitherto, the functional roles of FOXM1 and TYMS in the development of 5-FU resistance in *O. viverrini-*associated CCA have not been elucidated. To test this conjecture, we investigated the role of TYMS in 5-FU resistance and its regulation by FOXM1 and E2F1 in response to 5-FU in CCA.

RETRACTED

## Results

### A strong correlated overexpression of TYMS and FOXM1 in CCA tissues

Previous cDNA array studies have shown overexpression of FOXM1 mRNA in *O. viverrini*-associated CCA^11^. To investigate further the role and regulation of TYMS and FOXM1 in *O. viverrini*-associated CCA, the expression of TYMS and FOXM1 was determined by immunohistochemistry (IHC) in CCA tissue arrays. We found that FOXM1 expression was upregulated in 78% (88/113) and TYMS in 48% (54/113) of all *O. viverrini*-associated cases (*n* = 113) (Fig. 1; Supplementary Figs. S1, S2, S3). Notably, the results highlighted that FOXM1 is commonly overexpressed in CCA, suggesting its involvement in CCA tumorigenesis. This finding also suggested that the FOXM1–TYMS axis might have a wider role in tumour progression, such as chemosensitivity, as TYMS is a cellular target of 5-FU, the first-line chemotherapeutic drug for CCA.

**Fig. 1:** Correlation of FOXM1 and TYMS expression in CCA tissues. CCA tissue arrays were prepared from 113 *O. viverrini*-associated CCA cases using tissue microdissection techniques. **a** Representative immunohistochemical staining images showing correlated FOXM1 (top) and TYMS (bottom) expression. **b** Staining results and Chi-square analysis. Chi-square statistical analysis was used to test the correlations between TYMS and FOXM1 expression of CCA patients using GraphPad Prism 7.0 and and SPSS 16.0. In statistical analysis, *p < 0.05 was considered as significant

### Correlated baseline expression of FOXM1 and TYMS in CCA cell lines

To explore the relationship between FOXM1, E2F1 and TYMS expression and their functional roles in CCA, western blot and real-time quantitative PCR (qPCR) analyses were performed to determine the baseline steady-state expression levels of FOXM1 and TYMS, as well as one of their known regulator E2F1, in four CCA cell lines^25^. Consistent with the IHC results, western blot analysis revealed that in general FOXM1 was highly expressed and displayed good correlations with TYMS in CCA cells (Fig. 2a). Expression of E2F1 differed between the four cell lines and had little correlation with that of FOXM1 and TYMS, suggesting that FOXM1 and TYMS expression is not related to E2F1. Interestingly, TYMS expression was higher and FOXM1 expression lower in HuCCA compared to the other three CCA cell lines, KKU-D131, KKU-213 and KKU-214 (Fig. 2a). The mRNA levels of FOXM1, E2F1 and TYMS demonstrated good correlations with their protein levels in these CCA cells (Fig. 2b), indicating that the expression of these proteins are regulated primarily at the transcriptional level. Interestingly, the TYMS mRNA expression levels also demonstrated positive relationships with the FOXM1 in all but the HuCCA cell line, while E2F1 expression levels again did not appear to be associated with those of FOXM1 and TYMS in these CCA cell lines (Fig. 2b). Together, these results suggest that TYMS expression is regulated by FOXM1 but not by E2F1 in CCA cells. The discordance between FOXM1 and TYMS expression levels in HuCCA also suggests that TYMS expression is not coupled to FOXM1 regulation in this cell line.

RETRACTED

**Fig. 2:** Baseline expression of FOXM1, E2F1 and TYMS in CCA cells. CCA cells were harvested and the expression of FOXM1, E2F1 and TYMS at the translation and transcription levels were investigated using (**a**) western blot and (**b**) RT-qPCR. The latter assay was carried out in triplicate, and data are presented as means ± S.E.M. Expression of each gene was normalized relative to L19. The RT-qPCR data were analysed by one-way ANOVA with Fisher’s Least Significant Difference (LSD) post-test. Double and triple asterisks (** and ***) indicate significant difference at *p* < 0.01 and *p* < 0.001, respectively, from HuCCA (*n* = 3)

### HuCCA is a highly 5-FU-resistant CCA cell line

As TYMS is the direct cellular target of 5-FU, we next examined the four CCA cell lines, HuCCA, KKU-D131, KKU-213 and KKU-214, for their sensitivity to 5-FU using sulforhodamine B (SRB) assay. Viability of all CCA cell lines decreased in a dose-dependent manner after treatment with 5-FU after 24, 48 and 72 h; HuCCA remained the more resistant line compared with the other three and exhibited the highest IC50 (Fig. 3a; Supplementary Figs. S4, S5). We next examined the sensitivity of the CCA cells to 5-FU by clonogenic assays. Consistently, clonogenic assays revealed that HuCCA was the most resistant cell line (Fig. 3b; Supplementary Fig. S6). The results also showed that these CCA cell lines are relatively resistant to 5-FU treatment, consistent with the observations in the clinic that most CCAs are resistant to genotoxic chemotherapy^8–10^.

RETRACTED

**Fig. 3:** 5-FU treatment suppresses proliferation of CCA cells. CCA cells of HuCCA, KKU213, KKU214 and KKU-D131 lines were treated with different concentrations of 5-FU using DMSO as a vehicle. **a** Cell proliferation was assessed at 24, 48 and 72 h after 5-FU treatment using SRB assay. The experiment was carried out in triplicates and data are presented as means of the percentage of untreated control. The cell viability data were analysed by two-way ANOVA with Fisher’s Least Significant Difference (LSD) post-test (*n* = 3). The asterisks (***) indicate significant difference at *p* < 0.001. The IC50 for each CCA cell line at 48 and 72 h are shown (Supplementary Fig. S4). **b** The CCA cells were analysed for their sensitivity to 5-FU by clonogenic assays. After 48 h of incubation with the drugs, cells were cultured in fresh media, grown for around 14 days and stained with crystal violet. The graphs are representative of six experiments. Representative clonogenic images show the effects of 5-FU treatment (Supplementary Fig. S6). Data were analysed by two-way ANOVA with Fisher’s Least Significant Difference (LSD) post-test. The asterisk (*) indicates significant difference at *p* < 0.05. **c** Expression of FOXM1, E2F1 and TYMS in 5-FU-treated CCA cell lines in response to 5-FU. The CCA cell lines were treated with 100 µM of 5-FU over a period of 48 h. Cells were trypsinized at specific times and the expression of FOXM1, E2F1 and TYMS was determined using western blotting. β-Tubulin was used as a loading control. Representative western blot images are shown

### Coordinated FOXM1 and TYMS expression upon 5-FU-treatment in CCA cell lines

Since TYMS is an important target for 5-FU treatment and has previously been shown to be regulated by FOXM1 and E2F1, we therefore hypothesized that the expression levels of these proteins regulate 5-FU sensitivity. To test this conjecture, the four very 5-FU-resistant CCA cell lines were treated with a high dose of 100 μM 5-FU (see Fig. 3) over the course of 48 h, and the expression levels of FOXM1, E2F1 and TYMS proteins were examined by western blot analysis (Fig. 3c). Expression of FOXM1 in all four cell lines increased transient in a time-dependent manner and its expression level was the highest at 24 h posttreatment and declined thereafter, concomitant with a reduction in cell proliferation rates (Fig. 3a). This kinetics of FOXM1 expression is consistent with other cancer cells following treatment with genotoxic agents^13,22,26–29^. Similarly, the expression of TYMS mirrored that of FOXM1 but at a slower kinetics in the CCA lines, except for HuCCA where TYMS was expressed consistently at comparatively higher levels throughout the time course. The active metabolite of 5-FU, FdUMP, binds to TYMS to form an inactive slower migrating FdUMP–TYMS complex, which inhibits the conversion of dUMP to dTMP. Notably, using a high dose of 100 μM 5-FU to treat the CCA cells, the majority of the TYMS proteins were in the FdUMP-complexed inactive slower migrating (higher) forms following 5-FU treatment, and this lack of active unligated TYMS would lead to dNTP shortage and the cytotoxic DNA damage. Expression of E2F1 in all cell lines did not show good correlations with either FOXM1 or TYMS, indicating further that E2F1 does not control FOXM1 and TYMS expression or vice versa in response to 5-FU in these CCA cells. These results also further suggest that FOXM1 regulates TYMS expression in CCA cells, except for the resistant HuCCA.

RETRACTED

### Silencing of FOXM1 reduced the 5-FU resistance and TYMS expression in KKU-D131 but not in HuCCA cells

To further investigate the role of FOXM1 in modulating the sensitivity of 5-FU in CCA cells, western blot analysis was performed on the most sensitive KKU-D131 and resistant HuCCA cells in the presence and absence of FOXM1 depletion. The result revealed that TYMS expression decreased upon FOXM1 depletion using small interfering RNA (siRNA) in the sensitive KKU-D131 but not in the resistant HuCCA cells, suggesting that TYMS is, at least partially, regulated by FOXM1 in the sensitive but not in the resistant CCA cells (Fig. 4a). By contrast, FOXM1 knockdown did not cause any substantial changes in E2F1 levels in both cell lines, further confirming that FOXM1 does not regulate E2F1. Clonogenic assay was then performed to investigate the effects of FOXM1 depletion on 5-FU sensitivity in HuCCA and KKU-D131 cells (Fig. 4b). Silencing of FOXM1 did not overtly affect 5-FU sensitivity of the resistant HuCCA cell line but caused a decrease in the clonogenicity of KKU-D131 (Fig. 4b), suggesting that FOXM1 plays a significant role in modulating TYMS expression and hence 5-FU sensitivity in the sensitive but not in the resistant CCA cells. FOXM1 was next overexpressed in KKU-D131 and HuCCA cells. The control and FOXM1-overexpressing CCA cells were then tested for their sensitivity to 5-FU. Western blot analysis revealed that FOXM1 was overexpressed in the FOXM1-transfected KKU-D131 and HuCCA cells, and TYMS expression was not affected by FOXM1 overexpression (Fig. 5a). In concordance, clonogenic assay showed that ectopic overexpression of FOXM1 did not alter the sensitivity of either KKU-D131 or HuCCA cells to 5-FU (Fig. 5b). These results indicated that, although FOXM1 plays a vital role in the proliferation and 5-FU sensitivity of the KKU-D131, FOXM1 is already highly expressed and further overexpression would not induce additional TYMS expression and thereby 5-FU resistance. This notion is consistent with our earlier findings that FOXM1 is overexpressed in most CCA patient samples (Fig. 1) and cell lines (Fig. 2).

RETRACTED

**Fig. 4:** Effects of FOXM1 silencing on CCA cells in response to 5-FU treatment. FOXM1 expression in HuCCA and KKU-D131 cells was silenced using siRNA (siFOXM1) and non-silencing siRNA (NS-siRNA) was used as control. After 24 h, CCA cells were reseeded and grown overnight. **a** After treatment with 100 μM 5-FU for 24 h, cells were harvested and the expression levels of FOXM1, E2F1 and TYMS were determined by western blot and RT-qPCR analysis. Western blot was performed using β-tubulin as loading control (upper panel). Expression of FOXM1, E2F1 and TYMS mRNA was also determined by RT-qPCR analysis using L19 as an internal control (lower panel). Data are presented as mean ± SEM (*n* > 3). RT-qPCR data were analysed by unpaired *t* tests. Double and triple asterisks (** and ***) indicate significant difference at *p* < 0.01 and *p* < 0.001, respectively, from the non-targeting siRNA-treated control cells; ‘ns’ indicates no significant difference. **b** Effect of FOXM1 silencing on 5-FU sensitivity was also investigated using clonogenic assays. Representative clonogenic images show the effects of FOXM1 silencing on the outcome of 5-FU treatment. Data are presented as mean ± SEM (*n* = 3) and were analysed by two-way ANOVA. The asterisks (****) indicate significant difference at *p* < 0.0001 from the non-targeting siRNA-treated control cells; ‘ns’ indicates no significant difference

**Fig. 5:** Effects of ectopic expression of FOXM1 in KKU-D131 and HuCCA cells in response to 5-FU treatment. FOXM1 expression in KKU-D131 cells was induced by transfection with FOXM1-pcDNA3.1 plasmid DNA. Plasmid DNA from parental vector was used as transfection controls. After 24 h, CCA cells were reseeded and grown overnight. **a** After treatment with 100 μM 5-FU for 24 h, cells were harvested and the expression levels of FOXM1, E2F1 and TYMS was determined by western blot analysis using β-tubulin as loading control. **b** Effects of FOXM1 overexpression on 5-FU toxicity was also investigated using a clonogenic assay. Representative clonogenic assay images show the effects of FOXM1 overexpression upon 5-FU treatment. **c** Data are presented as mean ± SEM (*n* = 3) and were analysed by two-way ANOVA. No significant difference is indicated by ‘ns’

### Silencing of TYMS sensitizes both HuCCA and KKU-D131 cells to 5-FU treatment

In order to verify that TYMS expression is involved in the modulation of 5-FU sensitivity in CCA cells, TYMS expression was silenced using siRNA in both the 5-FU-resistant HuCCA and 5-FU-sensitive KKU-D131 cells, and the effects of TYMS knockdown on 5-FU sensitivity investigated using clonogenic assay. As shown in Fig. 6a, siRNA efficiently silenced the expression of the TYMS protein. Silencing of TYMS effectively sensitized both HuCCA and KKU-D131 to 5-FU, even at the lowest concentrations (e.g., 1 µM), confirming that TYMS is the target of 5-FU and its levels modulate 5-FU sensitivity in both the sensitive and resistant CCA cells (Fig. 6b; Supplementary Fig. S7). Unexpectedly, TYMS knockdown also resulted in a downregulation of FOXM1 expression (Fig. 6a), suggesting that TYMS might have a role in controlling the FOXM1 expression and FOXM1 as a sensor for TYMS activity and DNA damage, probably through the induction of DNA damage via blockage of replication fork progression. In addition, silencing of E2F1 by siRNA was also performed because expression of TYMS has previously been shown to be regulated by E2F1; however, E2F1 silencing did not affect the sensitivity of either HuCCA or KKU-D131 to 5-FU (Fig. 6b; Supplementary Fig. S7). Collectively, these data showed that TYMS expression levels determine the drug sensitivity in both sensitive and resistant CCA cells. In addition, the findings also supported the idea that FOXM1 regulates TYMS expression and thereby 5-FU sensitivity in CCA cells and that the uncoupling between FOXM1 and TYMS expression is linked to refractory to 5-FU in CCA cells.

RETRACTED

**Fig. 6:** Effects of E2F1 and TYMS silencing on 5-FU treatment of CCA cells. Either E2F1 or TYMS expression in HuCCA cell was silenced using siRNA (siE2F1 or siTS). Non-silencing siRNA (NS-siRNA) was used as a control. After 24 h, HuCCA cells were reseeded and grown overnight. **a** After treatment with 100 μM 5-FU for 24 h, cells were harvested and the expression of FOXM1, E2F1 and TYMS was determined by western blot analysis using β-tubulin as loading control. **b** Effects of E2F1 and TYMS silencing on 5-FU toxicity was also investigated using a clonogenic assay. Representative clonogenic assay images show the effect on 5-FU treatment of silencing of either E2F1 or TYMS. Data are presented as mean ± SEM (*n* = 3) and were analysed by two-way ANOVA. Single and triple asterisks (* and ****) indicates significant difference at *p* < 0.05 and *p* < 0.001, respectively, from the non-targeting siRNA-treated control cells; ‘ns’ indicates no significant difference

### FOXM1 modulates TYMS levels and 5-FU response in CCA cells

To further test the hypothesis that FOXM1 modulates 5-FU response through regulating TYMS expression levels in CCA, KKU-D131 and HuCCA cells were treated with a lower dose (20 µM) of 5-FU, which has differential cytotoxic effects on the comparatively more sensitive and resistant CCA cells (Fig. 7). As expected, in the comparatively more sensitive KKU-D131 both FOXM1 and TYMS protein and mRNA expression increased coordinately reaching a peak at 24 h posttreatment and decreased thereafter at 48 h. By contrast, despite the induction of FOXM1 expression in response to 5-FU in the resistant HuCCA cells, the expression of TYMS remained constantly high throughout the time course.

RETRACTED

**Fig. 7:** Expression of FOXM1, E2F1 and TYMS in CCA cell lines treated with a lower 20-µM dose of 5-FU. HuCCA and KKU-D131, the resistant and sensitive cell lines, respectively, were treated with 20 µM of 5-FU over a period of 48 h. Cells were trypsinized at specific times and the expression of FOXM1, E2F1 and TYMS was determined using western blotting. β-Tubulin was used as a loading control. **a** Expression of FOXM1, E2F1 and TYMS was determined by western blot analysis using β-tubulin as loading control. **b** Expression of FOXM1, E2F1 and TYMS mRNA was determined by RT-qPCR analysis using L19 as an internal control. Data are presented as mean ± SEM (*n* > 3). The RT-qPCR data were analysed by one-way ANOVA. The asterisk (*) indicates significant difference at *p* < 0.05

Critically, in the sensitive KKU-D131 cells the majority of the TYMS proteins were in the FdUMP-complexed inactive slower migrating forms especially after the coordinated downregulation of FOXM1 and TYMS expression at 48 h following 5-FU treatment, and this lack of active unligated TYMS would lead to cytotoxic DNA damage. By comparison, in HuCCA cells the levels of TYMS remained relatively stable over the time course with a substantial proportion remaining in the uncomplexed and active faster migrating species, and the cells could still be able to process the dUMP to dTMP conversion for DNA replication (Fig. 7).

### Differential binding of FOXM1 to endogenous TYMS promoter in 5-FU-sensitive and -resistant CCA cells

We next investigated the regulation of TYMS by FOXM1 at the promoter level. To this end, we first identified the putative FOXM1-binding regions from previously published FOXM1 chromatin-Immunoprecipitation–sequencing (ChIP-Seq) studies (Fig. 8). Both HuCCA and KKU-D131 cells were either untreated or treated with 5-FU for 24 and 48 h. To confirm further that FOXM1 binds to the endogenous *TYMS* promoter, we studied the occupancy of the endogenous *TYMS* promoter by FOXM1 using ChIP in the absence and presence of 24 or 48 h of 5-FU treatment in both cell lines. The ChIP analysis showed that FOXM1 is recruited to the endogenous Forkhead response element (FHRE) in both HuCCA and KKU-D131 cells and its binding to the FHRE increases substantially in KKU-D131 but not in HuCCA in response to 5-FU (Fig. 8; Supplementary Fig. S8). Together, these findings suggest that *TYMS* is a direct transcriptional target of FOXM1 in CCA cells and that the incapacity of FOXM1 to modulate TYMS expression is due its inability to be efficiently recruited by the promoter of *TYMS*.

RETRACTED

**Fig. 8:** Analysis of FOXM1 binding on human TYMS promoter **a** FOXM1-binding site on human TYMS promoter. ENCODE (the Encyclopedia of DNA Elements) project ChIP sequencing data of FOXM1 binding in the MCF-7, SKSH and ECC1 cells were used for predicting global genome-binding profiles for FOXM1 using the Integrative Genomics Viewer (Version 2.3.88) and the hg19 UCSC Genome Browser^50^. The predicted binding profiles of FOXM1 and the locations of the designed ChIP primer pairs are aligned to the human TYMS promoter. **b** KKU-D131 and HuCCA cells treated with 100 nM 5-FU for 0, 24 and 48 h were used for chromatin immunoprecipitation assays using the IgG as negative control and anti-FOXM1 antibody. After reversal of cross-linking, the co-immunoprecipitated DNA was amplified by qRT–PCR, using primers amplifying the FOXM1 binding-site-containing region. Data are presented as mean ± SEM (*n* = 4, each with >3 replicates) and were analysed by two-way ANOVA (Supplementary Fig. S7). The asterisk (*) indicates significant difference at *p* < 0.05 and ‘ns’ no significant difference

## Discussion

Surgery is the most effective treatment strategy for all potentially resectable intrahepatic CCAs^30^. However, owing to the late presentation and/or the advanced stages of most patients, CCA tumours are often not amenable to resection and chemotherapy. 5-FU either alone or in combination with other drugs is one of the most frequently used first-line regimens for CCA treatment. Nevertheless, the outcome is often sub-optimal because CCA patients are commonly intrinsic resistant or will become refractory after initial 5-FU treatment, leading to disease recurrence^8,31^. As TYMS is a key target of 5-FU, the possible mechanism of 5-FU resistance in CCA is likely to involve TYMS^16^ and its putative regulators FOXM1^14^ and E2F1^32^.

To test this conjecture, we first investigated FOXM1 expression by IHC in CCA tissue arrays and found that FOXM1 is highly expressed in almost all CCA cases, consistent with previously published mRNA expression profiling analyses^11,33^. FOXM1 has previously been shown to be a key genotoxic drug sensor and a regulator of chemotherapeutic resistance in cancer^13,15,26–29,34^. For instance, in breast cancer, FOXM1 expression is consistently higher in epirubicin (MCF-7^EpiR^) and cisplatin (MCF-7^CisR^) resistant cells compared to the parental sensitive breast cancer MCF-7 cells^13,22,28^. Moreover, drug treatment downregulates FOXM1 expression at both the transcriptional and posttranslational levels in the sensitive breast cancer, whereas FOXM1 expression remains at high levels in the resistant cells^13,22,26,27,29,34^. Furthermore, depletion of FOXM1 has been shown to sensitize breast cancer cells to genotoxic agents^13,22^. In agreement with this idea, high levels of FOXM1 expression have also been found to convey poor prognosis in breast cancer patients^13,22,35^. Taken together with these previous observations, our IHC led us to investigate the hypothesis that FOXM1 regulates TYMS to modulate 5-FU sensitivity. Notably, our finding that FOXM1 is overexpressed in almost all CCA cases (95%) is in concordance with previous observations that most CCAs are resistant to conventional chemotherapy^8,31^. However, owing to the lack of comprehensive clinical follow-up data and the late presentation of the patients, the correlations between FOXM1/TYMS expression and 5-FU sensitivity were pursued in CCA cell culture models and not in patient samples.

RETRACTED

In vitro clonogenic and proliferative studies showed that all CCA cell lines tested are highly resistant to 5-FU, consistent with the previous published CCA patient results^8,31^. These studies also identified HuCCA as the most 5-FU resistant among four human CCA cell lines (e.g., HuCCA, KKU-213, KKU-214 and KKU-D131). Western blot and quantitative reverse transcriptase PCR (qRT-PCR) analyses also unveil a discordance between FOXM1 and TYMS expression at the base line level in this highly 5-FU-resistant HuCCA line when compared with the other comparatively more sensitive CCA cells. Upon treatment with high doses of 5-FU, expression of FOXM1 in all four cell lines increased transiently in a time-dependent manner with the expression levels highest at 24 h and declined thereafter, concomitant with a reduction in cell proliferation and viability rates (Fig. 3). This kinetics of FOXM1 expression is analogous to those observed in drug-sensitive cancer cells upon genotoxic drug treatments, suggesting that FOXM1 is also a sensor for 5-FU induced DNA damage in CCA cells^13,22,26,27,29,34^. While FOXM1 and TYMS expression was coordinately modulated in response to 5-FU treatment in the 5-FU sensitive CCA cell lines, TYMS expression remained comparatively high throughout the time course in the resistant HuCCA cells, indicating a potential uncoupling between FOXM1 and TYMS expression in the resistant HuCCA cells. This conjecture is supported by our siRNA silencing analysis, which shows that FOXM1 depletion only reduces TYMS expression and 5-FU sensitivity in KKU-D131 but not in the highly resistant HuCCA cells. Based on the results, we conclude that TYMS expression is linked to 5-FU sensitivity, implying that TYMS overexpression plays a major role in 5-FU resistance. Consistent with this finding, previous studies have shown overexpression of TYMS as a 5-FU-resistance mechanism^36–38^.

RETRACTED

Notably, the 5-FU sensitivity and TYMS expression in HuCCA was not affected by FOXM1 silencing, suggesting that HuCCA is not sensitive to regulation by FOXM1. In concordance, ChIP analysis shows that in response to 5-FU, the binding of FOXM1 increases transiently before dropping to basal levels in the KKU-D131 cells but remains constantly low in the resistant HuCCA cells. These findings confirm that *TYMS* is a direct transcriptional target of FOXM1 in CCA cells and that FOXM1 fails to modulate TYMS expression in the resistant CCA cells because of its inability to be efficiently recruited to the *TYMS* promoter. This result is consistent with a recent FOXK1-ChIP-Seq analysis which shows the *TYMS* promoter contains FHRE^39^. The strong and significant correlations between FOXM1 and TYMS expression in CCA patient samples, further suggest that FOXM1 controls TYMS expression.

Time course experiments with a lower dose (20 µM) of 5-FU provide further evidence to support the notion that FOXM1 modulates TYMS expression levels and therefore 5-FU sensitivity in response to the drug. They also illustrate that the uncoupling of the FOXM1–TYMS axis allows a consistent level of unligated active TYMS to mediate DNA replication. This notion is supported by the fact that TYMS depletion by siRNA rendered the 5-FU resistance HuCCA cells sensitive to 5-FU treatment in clonogenic assays (Fig. 6). Our siRNA depletion studies also indicate that E2F1 is not involved in the regulation of TYMS and FOXM1 in CCA cells. In concordance, others have also found that TYMS is not regulated by E2F1 in other cell models^40^.

Interestingly, downregulation of FOXM1 was observed in TYMS knocked down HuCCA cell line. This observation might be explained by the fact that TYMS can suppress the 5-FU-induced DNA damage and expression of p53, which can in turn repress FOXM1 expression^41–43^. These results suggest that FOXM1 functions as a sensor of 5-FU-induced DNA damage and its regulation of TYMS determines 5-FU response in CCA. In agreement, FOXM1 has been shown to be a sensor of genotoxic agents and a modulator of their response. Accordingly, FOXM1 has been demonstrated to be regulated by SUMOylation and ubiquitination in response to genotoxic drug treatments and the ubiquitination-conjugating enzymes, RNF8 and RNF168, and the deconjugating enzyme OTUB1 play a crucial role in mediating this response by regulating FOXM1 expression at the posttranslational levels^27,29,34^.

RETRACTED

Interestingly, in contrast, overexpression of FOXM1 in both the 5-FU-sensitive and -resistant CCA cells does not affect TYMS expression nor 5-FU sensitivity, further confirming that in most CCA cells FOXM1 is already overexpressed at high levels. This observation is consistent with our IHC finding and previous gene expression profiling results^11,33^. FOXM1 overexpression could be a feature of CCA tumorigenesis, and therefore, FOXM1 and its gene transcription signature can be exploited as a useful biomarker for early CCA diagnosis. The mechanism for FOXM1 overexpression in CCA is unclear; however, exome sequencing has identified TP53 gene mutation as an event that may contribute to the initiation of *O. viverrini*-related CCA^44^. FOXM1, a gene highly expressed in CCA^11,33^, is one of the targets of p53-mediated repression^22,45^. Furthermore, the molecular mechanism of tumorigenesis for *O. viverrini*-associated CCA has been linked to inflammation-induced DNA damage^46,47^, and this could lead to the selection of p53-mutated and FOXM1-overexpressing CCA cells.

Collectively, our data provide evidence to show that FOXM1 regulates TYMS to modulate 5-FU sensitivity in CCA cells and that the high FOXM1 expression confers 5-FU resistance in most of these CCA cells through promoting high levels of TYMS expression (e.g., in KKU-M213, KKU-M214 and KKU-D131 cells). Moreover, we also found an alternative and novel mechanism for further 5-FU resistance, which is the uncoupling of the regulation of TYMS by FOXM1 (e.g., HuCCA). In support of the idea that the uncoupling of the regulation of TYMS by FOXM1 is uniquely important for 5-FU insensitivity in HuCCA cells, our preliminary data show that, despite HuCCA being the most resistant to 5-FU treatment among all the CCA cells tested, it is one of the more, if not most, sensitive to epirubicin and paclitaxel treatment (Supplementary Fig. S9). This is consistent with our previous finding that epirubicin and paclitaxel target DNA repair and mitotic genes via FOXM1 (e.g., NBS1 and KIF20A, respectively) to modulate their drug sensitivity^13,35^. Moreover, although overexpression of FOXM1 does not have any effect on 5-FU sensitivity in HuCCA, its ectopic expression can confer resistance to epirubicin and paclitaxel, respectively (Supplementary Fig. S10). These findings also propose the possibility of using alternative FOXM1-targeting cytotoxic agents to treat 5-FU-resistant cancer cells that have FOXM1–TYMS regulation uncoupled and lower FOXM1 expression.

RETRACTED

In conclusion, our results evidently show that FOXM1, but not E2F-1, modulates TYMS expression and thereby 5-FU sensitivity in CCA cells. Our data also demonstrate that the FOXM1–TYMS axis plays a major role in mediating 5-FU sensitivity in CCA cells and its uncoupling may be linked to 5-FU resistance. Our findings suggest the FOXM1–TYMS axis is a determinant of 5-FU response and a target for designing more effective treatment for CCA patients. Since FOXM1 is overexpressed in almost all CCAs and may be essential for CCA tumorigenesis, FOXM1 and its downstream transcriptional signature might also be useful for prognosis prediction of CCA.

## Materials and methods

### Chemicals and reagents

SRB and 5-FU were purchased from Sigma Aldrich (Irvine, UK). Rabbit anti-FOXM1 (C-20) and β-Tubulin (H-235) antibodies were from Santa Cruz Biotechnology (Santa Cruz, CA, USA). Rabbit anti-TYMS was obtained from Cell Signaling Technology (New England Biolabs Ltd. Hitchin, UK). Rabbit anti-E2F1 was purchased from Abcam (Cambridge, UK) and horseradish peroxidase (HRP)-conjugated secondary antibodies from Dako (Glostrup, Denmark) and Jackson ImmunoResearch (West Grove, PA, USA). Western Lightning® Plus-ECL was acquired from Perkin Elmer (PerkinElmer Ltd, Beaconsfield, UK) and SYBR Select Master Mix from Applied Biosystems (Fisher Scientific UK Ltd, Loughborough, UK).

### Human CCA cell lines

Four human CCA cell lines were used in this study. KKU-213 (mixed papillary and non-papillary CCA) and KKU-214 (well-differentiated CCA) were established from Thai CCA patients as described previously^17^. HuCCA was established from Thai patient with intrahepatic CCA^48^ and KKU-D131 CCA cell line was recently established from a Thai CCA patient. All cell lines were cultured in Dulbecco’s modified Eagle’s medium supplemented with 10% foetal calf serum (FCS) (First Link Ltd, Birmingham, UK), 2 mmol/L glutamine, 100 U/mL penicillin and 100 µg/mL streptomycin (Sigma-Aldrich, Poole, UK). All cell lines were maintained at 37 °C in in a humidified incubator with 10% CO_2_.

### IHC staining

IHC was performed as described elsewhere^49^. In brief, CCA tissue array slides were constructed at the Department Pathology, Faculty Medicine, Khon Kaen University, Thailand. All cancerous tissues were obtained from CCA patients who underwent surgery at Srinagarind Hospital, Khon Kaen Province, Thailand. All patients did not receive any chemotherapy prior to surgery. Tissue was deparaffinized and antigens were unmasked by autoclaving with sodium citrate buffer (10 mM sodium citrate, 0.05% Tween 20, pH 6.0). Thereafter, slides were immersed in 3% H_2_O_2_ for 10 min for endogenous peroxidase removal. Then non-specific binding was blocked by incubating with 5% FCS for 1 h at room temperature. Slides were then immersed with either rabbit anti-FOXM1 or TYMS (1:200) in 1% FCS overnight at 4 °C. After washing with phosphate-buffered saline (PBS) for 3 times, slides were incubated with 1:1000 HRP-conjugated secondary antibody for 1 h at room temperature. Immunoreactivity was developed by using 3,3-diaminobenzidine and slides were counterstained with Mayer’s haematoxylin. The expression was categorized as 0 = negative (either negative staining or positive <10% of CCA tissue area) and 1 = positive (positive staining >10% of the CCA tissue area) by 3 investigators and consensus scoring by at least two out of the three was chosen as definitive grading score.

RETRACTED

### Cell viability assay

Cell viability was investigated by SRB colorimetric assay. CCA cell lines were plated in 96-well plate at 2000 cells per well and incubated overnight. In the following day, CCA cell lines were treated with various concentrations of 5-FU in dimethyl sulphoxide (DMSO) for 24, 48 and 72 h. All plates were kept in humidified incubator at 37 °C and 10% CO_2_. Then cells were fixed with cold 40% (w/v) trichloroacetic acid and incubated for 1 h at 4 °C. After washing 5 times with slow running tap water, 100 μL of 0.4% SRB in 1% acetic acid was added and incubated at room temperature for 1 h. Then unbound dye was removed by washing with 1% acetic acid and left to air-dry overnight. Finally, SRB dye was dissolved with 10 mM Tris buffer and placed on a rotator for 30 min. The optical density at 492 nm were measured using the Sunrise plate reader (Tecan Group Ltd, Mannedorf, Switzerland).

### Clonogenic assay

CCA cells were seeded (1000 cells/well) in duplicate into 6-well plate. Then cells were treated with either vehicle (DMSO) or 5-FU for 48 h. Culture media was changed every 2 days without further treatment. For harvesting, media was removed and then colonies were washed with PBS and fixed with 4% paraformaldehyde for 15 min at room temperature. After washing with PBS for 3 times, colonies were stained with 0.5% crystal violet for 30 min. Finally, solution was removed and plates were washed with tap water for 5 times and left to dry overnight. Digital images of colonies were taken using digital camera.

### Cell transfection

For gene silencing, HuCCA and KKU-D131 were plated in at sub-confluent densities. The following day, HuCCA and KKU-D131 were transfected with ON-TARGET plus siRNAs (GE Dharmacon) targeting FOXM1, E2F1, or TYMS using oligofectamine (Invitrogen, UK) following the manufacturer’s protocol. Non-Targeting siRNA pool (GE Dharmacon) was used as transfection control. For gene overexpression study, either pcDNA3.1 plasmid DNA or pcDNA3.1-FOXM1 plasmid DNA were transfected into HuCCA or KKU-D131 using X-tremeGENE HP (Roche Diagnostics Ltd, Burgess Hill, UK) according to the manufacturer’s protocol. Cells were harvested at 24 h post-transfection for further experiment.

RETRACTED

### Western blot analysis

Protein was extracted from cell pellets using 2 volumes of RIPA buffer (50 mM Tris-HCl, 150 mM NaCl, 1% NP-40, 5 mM EDTA, 1 mM dithiothreitol, 1 mM NaF, 2 mM phenylmethylsulfonyl fluoride, 1 mM sodium orthovanadate) with protease inhibitor cocktail. Protein (20 µg) were separated by sodium dodecyl sulphate-polyacrylamide gel electrophoresis and then transferred to a nitrocellulose membrane. After blocking with 5% bovine serum albumin in Tris buffered solution with 0.05% Tween-20 (TBST, pH 7.5), membranes were incubated with primary antibodies overnight at 4 °C. After washing with 0.05% TBST, membranes were incubated with secondary antibodies and chemiluminescence reaction was developed using Western Lightning® Plus-ECL. β-Tubulin was used as loading control.

### RNA extraction, cDNA synthesis and real-time qPCR

mRNA was extracted from cell pellets using the RNeasy Mini Kit (Qiagen Ltd, Crawley, UK) and mRNA was reversed-transcribed to cDNA using the SuperScript III First-Strand Synthesis System (Invitrogen). Real-time qPCR analysis was performed in triplicate using SYBR Select Master Mix and specific primers (Supplementary Figure S11) according to the manufacturer’s instructions. The qRT-PCR conditions were as follows: 95 °C for 10 min for enzyme activation, followed by 40 cycles of denaturing at 95 °C for 3 s and primer annealing and cDNA amplification at 60 °C for 30 s. Relative gene expression was calculated and normalized by L19.

### Statistical analysis

Data are expressed as mean ± SD. Chi-square statistical analysis were used to test the correlations between TYMS and FOXM1 expression of CCA patients, respectively, using GraphPad Prism 7.0 (GraphPad Software Inc., La Jolla, CA, USA) and SPSS 16.0 (Imperial College London, Software Shop, UK); *p* < 0.05 was considered as statistically significant. For comparisons between groups of more than two unpaired values, analysis of variance was used, and *p* < 0.05 was considered as statistically significant.

## Supplementary information

Supplementary Figure Legends

Supplementary Figure S1

Supplementary Figure S2

Supplementary Figure S3

Supplementary Figure S4

Supplementary Figure S5

Supplementary Figure S6

Supplementary Figure S7

Supplementary Figure S8

Supplementary Figure S9

Supplementary Figure S10

Supplementary Figure S11
